The article "Novel application of anti‐human Fc nanobody for screening high‐producing CHO cells for monoclonal antibody" was published in 2022. Journal: Eng Life Sci.

# Novel application of anti‐human Fc nanobody for screening high‐producing CHO cells for monoclonal antibody

**DOI:** 10.1002/elsc.202200028

**Published:** 2022-08-23

**Authors:** Di Zhu, Zheng Wang, Yunxia Xu, Jing Lin, Mei Qiu, Jianghai Liu, Xinlei Li

**Affiliations:** ^1^ Chengdu Medical College Sichuan Province China; ^2^ ABLINK Biotech Co. Ltd. Chengdu China; ^3^ Shanghai Bao Pharmaceuticals Co. Ltd. Shanghai China

**Keywords:** Chinese hamster ovary cell, GFP, monoclonal antibody, nanobody, phage display

## Abstract

Animal‐derived anti‐IgG secondary antibodies are currently employed to stain and screen of human monoclonal antibody(mAb)‐producing cells, but using animal‐derived antibodies may raise the concerns of high cost, complicated operations and biological safety issues in biopharmaceutical manufacturing. Nanobodies(VHHs) are attractive forms of antibodies for their straightforward engineering and expression in both eukaryotic and prokaryotic systems. Using phage‐displayed immune llama VHH library, we identified new anti‐Fc VHHs that could bind to human Fc with high affinity. In GFP fusion format, the anti‐Fc VHH‐GFP generated dramatically stronger FACS signals than AF488 conjugated anti‐IgG antibodies when used for staining mAb‐producing CHO cells. Furthermore, preparative sorting of CHO cells based on anti‐Fc VHH‐GFP staining resulted in the enrichment of cell lines capable of synthesizing mAb at high productivity. This safe and cost‐efficient anti‐Fc VHH‐GFP may optimize the process of generating highly productive cell lines for therapeutic mAb production compared to conventional animal‐derived fluorescent antibodies.

**Abbreviations**
AF488: Alexa Fluor 488
BSA: bovine serum albumin
ELISA: enzyme‐linked immunosorbent assay
FACS: fluorescence‐activated cell sorting
FBS: fetal bovine serum
Fc: crystalline fragment
FW: framework
GFP: green fluorescent protein
IgG1: immunoglobulin G1
IPTG: Isopropyl β‐D‐1‐thiogalactopyranoside
mAb: monoclonal antibodies
MSX: methionine sulfoximine
PBMC: peripheral blood mononuclear cells
scFv: single‐chain variable fragment
TMB: 4,4′‐Diamino‐3,3′,5,5′‐tetramethylbiphenyl
VHH: variable domain of the heavy‐chain of heavy‐chain antibody

## 1 INTRODUCTION

The screening and enrichment of high‐producing cells remains a great challenge in manufacturing monoclonal antibodies (mAb) [1, 2, 3]. The traditional limited dilution method is mature and reliable, but it is time‐consuming and has a low throughput process [4, 5]. The main problem is that high producers spend much cell energies on production, and thus have reduced growth rate, which leads to rare portion of desired clones outgrown by non‐ or low‐producing cells [6, 7]. Hence, an efficient and high throughput selection method is even more important. In recent years, with the development of technology, novel single cell screening methods have been developed to facilitates more efficient isolation of clonal cells with high productivity, such as new single cell analysis and separation systems including microfluidic technology and Beacon platform [8], label‐free screening methods based on cell surface display technology [9], Clonepix analyzing cells grown in semi‐solid and picked by clonal fluorescence microscopy [10].

Previous findings that secreted proteins would be transiently trapped on the cell surface and correlate with the amount of proteins being secreted from the cell, shed light on the use of flow cytometry and cell sorting to isolate a rare high‐producing cell [11]. Fluorescence‐activated cell sorting (FACS) classifying cells based on the determined fluorescence levels has been proven to be efficient and liable [12]. However, a fluorescent anti‐IgG antibodies used in the screening process are all animal‐derived, leading to the concerns about the biological safety in biopharmaceutical manufacturing [13]. Therefore, we aimed to seek for a recombinant antibody for cell labeling and selection for high‐producing subclones from transfected cell pools. Studies have shown that the fusion antibody of single‐chain variable fragment (scFv) and green fluorescent protein (GFP) allows direct labeling of cells in flow cytometry, avoiding the loss of antigen binding ability and reducing the background staining [14, 15]. In 1993, scientist Hamers‐Casterman first reported the presence of antibodies naturally lacking the CH1 domain and light chain (namely VHH or Nanobody) in camel blood [16], marking a new era of antibody engineering. Compared to scFv, VHH has more advantages in structural stability, small molecular weight, expression yield, ease of DNA manipulation and library construction [17, 18].

In this study we used VHH‐GFP against to human immunoglobulin G1 (IgG1) Fc fragment to select for high‐producing subclones of a recombinant CHO cell line producing a human antibody against Her2. The anti‐Fc VHH was screened by phage display, fused with GFP and produced at large scales in *E. coli*. The purified VHH‐GFP was used to label CHO cells and isolate the high producers using fluorescence intensity as a criterion. At last, the expression levels of anti‐Her2 mAb in different subclones were measured. The feasibility of VHH‐GFP in cell sorting for higher producers was evaluated by comparison with the conventional fluorescent antibody (Goat anti‐human IgG (H+L) antibody, Alexa Fluor 488).

**PRACTICAL APPLICATION**

Anti‐Fc VHH‐GFP fusions reported here is the first nanobody that are employed to screen high‐yielding CHO for monoclonal antibody. Compared to traditional AF488 conjugated anti‐human IgG antibodies, preparative sorting of cells based on VHH‐GFP staining has increased mAb‐expressing levels after further culture. The results of this study can provide scientific references for screening of transfected CHO cells with high productivity.

## 2 MATERIALS AND METHODS

### 2.1 Human Fc domain expression

The open reading frame of the human IgG1 Fc domain was obtained through total gene synthesis. The plasmid was digested with endonucleases *Eco*RI and *Bsi*W1(Thermo) to produce sticky ends, which was purified from agarose gel (Tiangen Biochemical Technology Co., Ltd.). The human IgG1 Fc fragment amplified by PCR was subcloned into a linearized eukaryotic expression vector (pFcIG) with secretion signal peptide and transformed into *E. coli* Trans5α, which was screened by ampicillin. Monoclonal sequencing (Qingke Biotechnology Co., Ltd.) was performed the next day, and the sequencing results were blasted with the expected sequence. Next, we amplified and cultured the host bacteria containing the recombinant plasmids. According to the manufacturer's instructions, we obtained endotoxin‐free plasmids using the Endotoxin Removal Kit (Tiangen Biochemical Technology Co., Ltd.). Cell density (293F) was adjusted to 6 × 10^5^ mL^–1^ by adding medium OPM‐293 CD05(shanghai OPM Biosciences CO., Ltd). Then the IgG1 Fc recombinant plasmid was mixed with suspension cell transfection reagent FectoPRO (Polyplus Transferion® SA), then transfected into HEK293F. After 5 days of shaking, the cells were incubated at 37°C, 220 rpm and 5% CO_2_. The supernatant was collected by centrifugation at 500 g for 3 min. The recombinant human lgG1 Fc protein was purified using Protein A resin (Genscript Biotech Corporation).

### 2.2 The immunization within alpaca

Two alpacas were injected with human IgG1 Fc recombinant protein subcutaneously and intramuscularly on the back of the neck to form multiple masses. The absorption of subcutaneous injection masses was followed up to confirm the correct immunity. The alpaca was immunized by four consecutive injections with an interval of 21 days. The antigen of each immunization was mixed with adjuvant (Sigma–Aldrich) in an equal volume ratio to form a stable emulsion. Antigen (0.5 mg) with Freund's Adjuvant Complete was used for the first immunization, and antigen (0.25 mg) with Freund's Adjuvant Incomplete was applied to all subsequent immunizations. A blood sample (10 mL) was collected before immunization as a control. A blood sample (50 mL) was collected and placed in a sterile vacuum tube, filled with lithium heparin to prevent blood clotting 1 week after the last injection. After immunization, an enzyme‐linked immunosorbent assay (ELISA) was used to measure the serum titer against the Fc domain of human IgG1 to monitor the immune. The results of ELISA showed that the titer of alpaca serum is > 1:32000, indicating that there is a high‐affinity antibody against human IgG1 Fc in the serum.

### 2.3 Library construction

Peripheral blood mononuclear cells (PBMC) were isolated from blood samples using ficoll‐hypaque (TBD) density gradient centrifugation, and centrifuged twice with 10 mL of saline at 4°C for 8 min at 500 g. Then, they were resuspended with 2–3 mL of saline and counted. PBMC (2 × 10^7^cells/tube) were taken for total RNA extraction, and the remaining cells were added to cell freezing solution including 90% fatal bovine serum and 10% DMSO in separate tubes at ‐80°C. Total RNA was extracted from PBMC using the High Purity RNA Isolation Kit (Foregene Co., Ltd.) according to the instructions. Total RNA (3∼5 μg) was taken for cDNA synthesis using RT‐PCR kit (Takara) with oligo(dT) as a primer.

The sequences of IgG2 and IgG3 heavy chain variable regions were amplified by nested PCR as follows: The cDNA was used as the template for the first round of PCR amplification. The nested outer primers were located in the heavy chain signal peptide region and the highly conserved region of the CH2 structural domain, and designed to amplify the alpaca heavy chain antibody gene fragments, the VH‐CH1‐CH2 fragment of size 900 bp and the VH‐CH2 fragment of about 700 bp, respectively. The 700 bp PCR product was cut by DNA gel electrophoresis, and then purified using a PCR product purification kit (Tiangen Biochemical Technology Co., Ltd.). Using the 700 bp product as a template, a second round of PCR was performed using the inner primers located within the Framework 1(FW1) and Framework 4 (FW4) to amplify the heavy chain antibody variable region (VHH fragments) of approximately 400 bp. VHH was subcloned into the linearized phage vector Pshort digested by *Eco*RI and *Xba* I by Gibson Assembly ligation reaction. The recombinant plasmid was transferred to *E.coli* SS320 containing the helper phage M13K07. After transformation, the bacterial broth was resuspended in SOC medium and activated in 37°C shaker for 1 h. The appropriate dilution titer was dropped on plates containing LB media supplemented with carbenicillin, incubated at 37°C overnight in a biochemical incubator for the calculation of library capacity and colony PCR identification. The remaining broth was transferred to a large volume of 2YT supplemented with carbenicillin, then placed in 37°C shakers overnight incubation. From this medium, the supernatant was harvested the next day, and 1/4 volume of PEG/NaCl (20% PEG/2.5 M NaCl) was used to precipitate the phage from the supernatant. The precipitation was repeated to remove bacterial cells, and the phage library was resuspended to obtain a phage display immune antibody library (stored at ‐80°C for later use).

### 2.4 Enrichment of anti‐human Fc VHH phages through panning

Human IgG1 Fc recombinant protein (5 μg/mL) was added to 96‐well plate (100 μL/well) and incubated at 4°C overnight. *E. coli* NEB5αF' was streaked and cultured overnight on plates at 37°C in the incubator. Single clones were picked from the plate and added to 2YT. The bacteria were shaken at 37°C until the value of OD_600_ was up to 0.8. At the same time, the antigen supernatant of the 96‐well plate was removed. Bovine serum albumin (1% BSA, 200 μL) was added to antigen wells and negative control wells. The plate was placed on a 3D rotary shaker at room temperature for 2 h. The supernatants of protein wells and control wells were washed with 200 μL PT (PBS buffer containing 0.05% Tween‐20), and 100 μL phage antibody library was added, respectively. The plates were placed on a 3D shaker at room temperature for 2 h. Then weakly bound phages or excess phages were washed away by PT. The target phage was eluted with 100 μL 100 mM HCl at room temperature for 5 min. The supernatant was pipetted out, transferred to a 1.5 mL centrifuge tube and neutralized with 1 M Tris‐HCl buffer. The mixture was added to a centrifuge tube containing 1 mL of NEB5αF' bacteria and incubated on a shaker for 1 h at 37°C 220 rpm. Bacteria from the centrifuge tube were diluted at an appropriate ratio and dropped on the plate. The plate was placed in a 37°C biochemical incubator overnight, and the titer and enrichment score was calculated next day. The remaining culture was incubated with 1 L of auxotroph M13K07(final concentration of 10^10^ mL^–1^) for 1 h at 37°C on a shaker at 220 rpm; the bacteria mentioned above were transferred to 35 mL of 2YT, placed on a shaker, and cultivated overnight at 37°C. Meanwhile, phages were collected to form an antibody library for each round. The above process needs to be repeated for 3∼5 rounds until phage enrichment is achieved.

### 2.5 Phage ELISA and clone sequencing

The 400 μL 2YT was added to each well in a 96 deep well plate. A single clone was picked from the enriched LB culture plate and amplified. The supernatant was obtained by centrifugation the next day containing the phage produced by each clone. Meanwhile, the recombinant human IgG1 Fc protein was diluted to 1 μg/mL and coated on a 96‐well ELISA plate at 4°C overnight.PVA (1%) was added to each well to prevent other proteins from adsorbing due to electrostatic or hydrophobic effects, which will lead to false‐positive signals and interfere with subsequent experiments. Besides, 1% PVA was added to the blank wells as a negative control. After 2 h of blocking at room temperature, the antigen and negative control wells were washed with PT solution. The supernatant (50 μL) from the 96 deep well plate was added to each well and incubated for 2 h at room temperature. After binding, the ELISA plate was washed with PT solution. Then 100 μL of anti‐M13 HRP antibody (Sino Biological Inc.) was added and the plate was incubated at room temperature for 1 h. At the end of washing sequentially with PT solution and PBS solution, 100 μL TMB (Shanghai Solarbio Bioscience & Technology Co., Ltd.) was added and incubated for 5 min at room temperature, and 50 μL 1 M phosphoric acid was added to terminate the reaction. The absorbance was measured at 450 nm with an enzyme‐labeled instrument. If the OD value > 4, the enzyme‐labeled instrument will display overflow. The single clones corresponding to the antigen well with OD > 0.5 and the negative control well with OD < 0.2 were identified as positive clones with higher affinity, and the monoclonal DNA sequencing was performed.

### 2.6 Nanobody recombinant protein expression and purification

The fully synthesized TAT‐GFP fragment was cloned into pET25b(+) plasmid through restriction sites *Xho* I and *Bam*HI, and transformed into *E.coli* trans5α, screened by ampicillin. Three single clones were randomly selected and sequenced to obtain the correct recombinant plasmid pTAT‐GFP.

VHH‐his and VHH‐GFP were expressed in *E.coli*. The positive clones 1 and 16 obtained by ELISA were selected for PCR, subcloned into the linearized vector PTAT‐GFP/PET‐25b(+) digested with *Bam*HI and *Xho* I, electrically transferred to the *E. coli* for expression. The transformed bacteria were incubated overnight at 37°C, 220 rpm in 2YT added ampicillin until the absorbance at 600 nm reached 0.6∼0.9. The VHH expression was induced overnight at 18°C by adding 0.5 mM IPTG (Biochemicals). Then the cells were collected and resuspended in PBS, lysed with Sonicator, and the supernatant was collected. After that, the supernatant was centrifuged at 4°C, 12000 rpm for 20 min to remove bacterial debris. GFP‐VHH‐His fusion protein was obtained after purification by immobilized metal ion affinity chromatography. The purity of the recombinant protein was evaluated by SDS‐PAGE (15% acrylamide) and stained by Coomassie brilliant blue to assess the purity of VHH‐GFP.

VHH‐mFc (mouse IgG2a Fc) was expressed in 293F cells. The experimental method is the same as the human Fc domain expression method.

### 2.7 Antibody conjugated to Alexa Fluor 488

The VHH‐his and VHH‐mFc was conjugated with Alexa Fluor 488 dye according to the manufacturer's instructions (Protein Labeling Kit A30006, Thermo). For the conjugation, the antibody was reconstituted in sodium bicarbonate and mixed with the dye as recommended by the manufacturer. The antibody‐dye mixture was incubated for 45 min at room temperature. Unconjugated dye was removed with centrifugation on an ultrafiltration column. After that, the fluorophore:VHH ratio of the labeled antibodies was calculated.

### 2.8 Affinity determination

Human IgG1 Fc protein (2 μg/mL) was coated onto the wells of 96‐well ELISA plate at 4°C overnight. The blocking solution was coated as a negative control. Then wells were blocked by 1% PVA and incubated with VHH‐GFP (1 and 16) for 2 h at room temperature. After two times of wash, the bound VHHs were detected by the secondary antibody to the alpaca IgG VHH domain conjugated with horseradish peroxidase(HRP). Peroxidase activity was measured at 450 nm after the addition of TMB as a substrate.

### 2.9 Detecting fluorescence value by flow cytometry

Jurkat cells were collected to be centrifuged at 500 g for 5 min, and washed 3 times with an appropriate amount of 4°C pre‐cooled PBS buffer. Cell suspension (5 × 10^5^ cells) was added to each flow assay tube and centrifuged. Then 100 μL of 10 μg/mL anti‐CD3 nano‐antibody (h20‐hFc) was added and incubated for 1 h in the refrigerator. After incubation was complete, the cells were washed by pre‐chilled PBS buffer three times to wash away unbound primary antibodies. VHH‐GFP (100 μL) was added to each tube and placed on ice for 1 h in the dark; then the supernatant was removed after centrifugation at 500 g for 5 min. After washing with PBS 3 times, the fluorescence value was measured by flow cytometry.

The stable cell line with high production of anti‐Her2 IgG1 monoclonal antibody was derived from Shanghai Baoji Pharmaceutical Co., Ltd. Positive cells (the stable cells) and negative cells (untransfected cells) were mixed at the ratio of 1:1. Mixed cells (0.5 × 10^6^)were washed with PBS and centrifuged at 1000 rpm for 5 min. Blocking solution (CD‐CHO medium from GIBCO containing 1% Human Serum Albumin, HSA) was added for resuspending. Then the cells were placed in the 37°C incubator for 60 min. Cells were mixed every 5∼10 min to prevent the cells from adhering to the wall. After blocking, cell density was adjusted to 2.5 × 10^6^ cells/mL and stained for 30 min at 4°C in the dark by different fluorescent antibodies (50 μg/mL) respectively, including VHH‐1/16‐GFP, the traditional fluorescent secondary antibody (AF488 conjugated goat antibody), AF488‐tagged VHH, and AF488‐tagged VHH‐mFc fusion protein (VHH‐mFc‐AF488). The stained cells were washed and resuspended in 200 μL PBS, then filtered through a 40 μm filter to remove clumps and detected for flow cytometry.

### 2.10 Stable CHO cells expressing IgG1

CHO K1 has been adapted to serum‐free and suspension culture conditions and is therefore used as the host cell. Cells for transfection were cultured in CD‐CHO (GIBCO) medium supplemented with 1 mM alanyl‐glutamine (Sigma–Aldrich) and placed on a shaker at 37°C with 5% CO_2_. The DNA sequence corresponding to recombinant humanized anti‐Her2 monoclonal antibody (*r*hHER2‐mAb) was designed, synthesized, and then cloned into the expression vector to construct the recombinant expression plasmid. CHO‐K1 cells (4.5 × 10^6^) were transfected by 4 μg plasmid, resuspended with pre‐warmed CD‐CHO medium at 5 × 10^5^ cells/mL, and cultured statically at 37°C, 5% CO_2_. After 48 h transfection, methionine sulfoximine (MSX, Sigma–Aldrich) was added to the culture medium. Centrifugation was performed every 2 days, and the CD‐CHO medium containing a certain concentration of MSX was added. After 4 days of transfection, the cell pool resistant to the corresponding antibiotic concentration was obtained.

The cell sorting was carried out by F.sight. A roundness was set from 0.6∼1, FL intensity was 80 mW, and exposure time was 10 ms for sorting. Subcloning medium 100 μL containing 5 μM MSX and 1% Fetal Bovine Serum (FBS)was added to each well in a 96 well plate, then another 100 μL medium was added after 7 days. The culture was carried out at 37°C and 5% CO_2_ at 120 rpm/min. The clone formation rate was determined every other week. When the clone formation rate was up to 60%, protein concentration was quantitatively monitored using Forte Bio during cultivation.

## 3 RESULT

### 3.1 Phage display selection of VHH specific for human IgG1 Fc

In order to generate VHH specific for human IgG1 Fc, the llama received four doses of the purified human IgG1 Fc protein. ELISA was used to monitor the serum antibody titer, which reached 1:128000 after the fourth dose. Then lymphocytes from the peripheral blood of immunized camels were separated, and the total RNA extracted was reverse transcribed into cDNA. The heavy chain variable regions of IgG2 and IgG3 were amplified using the cDNA template and cloned into M13‐based phage. After transforming the recombinant phage into super competent cells SR320 with helper phage, a VHH phage library containing 4.57 × 10^9^ clones was generated.

During the biopanning process, two rounds of in vitro selection were performed using immobilized human IgG1 Fc as an antigen. Antigen‐specific phages were enriched. Then 32 single clones were randomly selected for phage ELISA verification. All of these showed high affinity to human IgG1 Fc antigen (Figure 1). Seventeen colonies were randomly selected and sequenced. The complementarity determining region (CDRH1 and CDRH2) of VHH clones showed limited diversity in length and sequence, but the CDRH3 of VHHs is highly variable [19].

**FIGURE 1:** The capacity of the phage clones to bind human IgG1 Fc (5 μg/mL) or PVA

### 3.2 Characterization of the affinity of VHH‐1‐GFP and VHH‐16‐GFP with human IgG1 Fc domain

Two clones_,_ namely VHH‐1 and VHH‐16, were subcloned into the expression vector pTAT‐GFP providing a carboxy‐terminal His_6_ tag and produced in *E. coli*. After purification by immobilized metal ion affinity chromatography, the yield of proteins is up to 100∼150 mg/L. The molecular weight of VHH‐1‐GFP and VHH‐16‐GFP (45KD) were verified by SDS‐PAGE and showed more than 90% purity by SDS‐PAGE. In addition, VHH‐1‐GFP and VHH‐16‐GFP strongly recognized the immobilized human IgG Fc protein as determined by ELISA, with the EC50 of 0.27 nM and 0.29 nM, respectively (Figure 2).

**FIGURE 2:** (A) SDS‐PAGE profile of recombinant anti‐human Fc VHH after Ni‐column purification. (B) Two unique VHHs obtained from the panning were tested for binding affinity to human IgG1 Fc protein. Antibodies were incubated at room temperatures for 1 h, and then assayed in the standard human lgG1 Fc domain‐specific ELISA. The EC50 of VHH‐1‐GFP and VHH‐16‐GFP were 0.27 nM and 0.29 nM respectively

### 3.3 Staining of Fc domain at the cell membrane with anti‐Fc VHH‐GFP

We have investigated the capability of VHH‐GFP to label the cell surface protein. CD3‐expressing jurkat cells were first incubated with the primary antibody h20‐hFc (a human anti‐CD3 VHH fused with Fc domain), and then stained with 1 μg/well VHH‐1‐GFP or VHH‐16‐GFP. Cells treated with VHH‐GFP only were the negative control. Flow cytometry results showed that cells treated with h20‐hFc and then VHH‐GFP demonstrated a significant increase of fluorescence intensity compared with the negative control (Figure 3). The results suggest the specificity of VHH‐1‐GFP and VHH‐16‐GFP to detect the Fc domain bound on the cell surface.

**FIGURE 3:** The binding activity of VHH‐GFP by flow cytometry. (A) 5.5 × 10^6^ Jurkat cells were incubated with h20‐hFc, and then 1 μg VHH‐1‐GFP (grey curve). (B) 5.5 × 10^6^ Jurkat cells were incubated with h20‐hFc, and then 1 μg VHH‐16‐GFP (grey curve). The black curve represents negative control cells that were incubated with VHH‐GFP only

### 3.4 Staining of secreted mAb at the cell membrane with anti‐Fc VHH‐GFP

As secreted antibodies were transiently present on the cell surface, the antibody‐expressing cells can be stained with fluorescent secondary antibodies, and this antibody‐specific staining can be also used as the basis for flow cytometry sorting [8]. To further examine the ability of VHH‐GFP to discriminate mAb‐expressing and non‐expressing cells, CHO cells stably expressing human anti‐Her2 mAb were mixed with untransfected cells at 1:1 ratio. The mixture was probed with different fluorescent antibodies, including VHH‐1/16‐GFP, the traditional fluorescent secondary antibody (AF488 conjugated goat antibody), AF488‐tagged VHH, and AF488‐tagged VHH‐mFc fusion protein (VHH‐mFc‐AF488).

We first labeled VHH and VHH‐mFC(mouse IgG2a Fc) with organic fluorophores AF488. However, flow cytometry data showed that no staining was seen in this case (Figure 4B,C). This was presumably due to the change of the spatial structure of the antigen binding region (CDR) of VHH after conjugation with AF488. VHH‐AF488 fused with mouse IgG2a Fc (VHH‐mFc‐AF488) gave intense signals, but also the strong background, which would interfere with selection of mAb‐expressing cells (Figure 4D,E). In this experiment, three antibodies, AF488 conjugated goat antibody, VHH‐1‐GFP, and VHH‐16‐GFP could clearly distinguish between negative and positive cell populations (Figure 4A,F,G). VHH‐1‐GFP staining showed the highest MFI value for mAb‐expressing cells. Therefore, VHH‐1‐GFP were selected for further flow cytometry sorting.

**FIGURE 4:** Staining cell surface mAb with different fluorescent secondary antibodies by flow cytometry. Positive cells (the anti‐Her2‐mAb expressing CHO cells) and negative cells (non‐expressing cells) were mixed at the ratio of 1:1. The mixed cells were incubated with (A) Alexa Fluor 488‐conjugated goat anti‐human IgG (H+L) antibody (gray line), (B) Alexa Fluor 488‐tagged VHH‐1 (gray line), (C) Alexa Fluor 488‐tagged VHH‐16 (gray line), (D) Alexa Fluor 488‐tagged VHH1‐mFc, (E) Alexa Fluor 488‐tagged VHH16‐mFc, (F) VHH‐1‐GFP, (G) VHH‐16‐GFP or PBS (black line) for 30 min

### 3.5 High throughput screen of high‐producing CHO cell lines with anti‐Fc VHH‐GFP

Cells were further sorted based on the level of mAb associated with the cell surface. CHO‐K1 cells was transfected by electroporation with the anti‐HER2 mAb‐expression plasmids. After 4 days of selection and culture, the cell pool with a variety of different mAb expression levels were obtained. Cells stained by VHH‐1‐GFP or AF488 conjugated goat antibody were sorted by F. sight, which can efficiently and sensitively separate cells based on the different fluorescence intensity, as well as the cell size and roundness [20]. VHH‐1‐GFP staining showed dramatically higher fluorescence intensity than that stained with AF488 conjugated goat antibody (Figure 5A,B). The fluorescence value of single cells was also shown in Figure 5C. For preparative sorting, a gate was set which encompassed cells with the top 30% the fluorescence intensity, and larger than 12 μm with a roundness of 0.6∼1 to exclude non‐viable and irregular‐shaped cells. Sorted cells subsequently collected and expanded at 1 cell/well into 96‐well plates under selective conditions.

**FIGURE 5:** Sort of highly‐expressing cells from a transiently‐transfected cell pool by F.sight. The unstable cells were stained by (A) Alexa Fluor 488‐conjugated human IgG (H+L) antibody, (B) VHH‐1‐GFP for 30 min, then the cell size and fluorescence intensity were measure by F.sight. (C) Fluorescence intensity line profiles for cells stained with different secondary antibodies

### 3.6 Generation of high‐expressing recombinant CHO cells

All cloning plates were analyzed for antibody expression 20‐day post‐plating, when 60% subclones were successfully formed. The concentration of anti‐Her2 mAb of each subclones was quantitatively measured by ForteBio. The average mAb concentration for subclones sorted by VHH‐1‐GFP was 15.75 mg/L, and the maximum value was 28 mg/L, while the average value of subclones screened by AF488 conjugated goat antibody was 9.14 mg/L, the highest value was 17.8 mg/L (Figure 6). These data confirmed that VHH‐1‐GFP can be used for flow cytometry sorting to efficiently enrich high mAb‐expressing CHO cells.

**FIGURE 6:** Evaluation of anti‐Her2 mAb concentration of cells sorted by Alexa Fluor 488‐conjugated secondary antibodies or VHH‐1‐GFP. The subcloning medium was pressurized with 5 μM MSX and supplemented with 1% fetal bovine serum. Cells were cultured in 96‐well plates at 37°C, 120 rpm/min and 5% CO_2_ for 20 days

## 4 DISCUSSION

Chinese hamster ovary cells have become the most important cell lines for industrial production of therapeutic mAb drugs due to their widely proven safety and similar glycosylation modifications to human proteins [21]. To select rare high mAb‐expressing cells from transfected pools, the FACS‐based method by measuring the level of cell surface associated mAbs has been established as a robust and convenient screening strategy [8]. The recombinant cell lines is usually stained by fluorescently‐labeled antibodies derived from animals. However, using animal‐derived antibodies may raise the concerns of high cost, complicated operations and biological safety issues in biopharmaceutical manufacturing. In this study, our goal is to find a good substitute for traditional fluorescence antibodies to enrich high‐producing cells.

Nanobody is an idea candidate for detection reagents. It has been shown that VHH‐based detection reagents can improve the sensitivity of detection and shorten the detection and analysis time of ELISA and Western blot [22, 23, 24]. VHH not only preserve the binding affinity and specificity of the original whole antibody, but are appreciated for their smaller size, structural stability and easy preparation. The smaller size facilitates DNA manipulation and library construction. Nanobodies have been expressed in microbial systems with high yield but short production time. In the current study, the yield of VHH‐1‐GFP and VHH‐16‐GFP is up to 100∼150 mg/L of culture and the purity is estimated to be about 90%. Traditional fluorescent secondary antibodies are mostly animal‐based production. Because of the absence of more sustainable alternatives in the past, a continuous supply of anti‐IgG sera is required, which is not only costly but also raises animal welfare concerns [25]. In addition, each new batch of serum contains another heterogeneous mixture of antibodies and animal‐derived virus, requiring laborious quality control efforts. But small batch‐to‐batch variation from prokaryotic expression is easy for large‐scale production. Therefore, the production of VHH in prokaryotic expression usually gives high yields, low time‐ and labor‐cost, and avoidance of microbial contamination.

In the current work, we employed fluorescent labeled anti‐Fc VHH to discriminate mAb‐expressing and non‐expressing cells. We first labeled VHH and VHH‐mFc (mouse IgG2a Fc) by chemical conjugation of organic fluorophores AF488. Flow cytometry results suggest that bound fluorochromes may result in partial or complete loss of antigen‐binding capacity, presumably because conjugation occurs within the antigen‐binding sit (Figure 4B–E). However, anti‐Fc VHH‐GFP fusions can successfully label the cells secreting mAbs and distinguish between negative and positive cell populations (Figure 4F,G). Moreover, VHH‐GFP fusions has several advantages over its fluorescent conjugation form from the handling point view. Firstly, GFP is a non‐invasive protein and VHH‐GFP can be expressed in bacteria with high yield [26]. Secondly, the recombinant protein (VHH‐GFP) is always represented in a one‐to‐one ratio between fluorescent dye and target proteins, which improves the accuracy of quantitative analysis [27, 28].

The effectiveness of anti‐Fc VHH‐GFP to isolate and enrich cells producing high mAb levels was tested on CHO cell pools producing a human antibody against Her2. The results of F.sight analysis showed that the cells stained with VHH‐1‐GFP demonstrated stronger fluorescence values than traditional fluorescent secondary antibodies (Figure 5A,B). Our explanation was that the smaller molecular size and longer CDRH3 region enables VHH‐1‐GFP recognition of epitopes not easily accessible by traditional fluorescent secondary antibodies and production of an increased signal. Moreover, the number of monoclonal cells with fluorescence intensity greater than 100 is 14 times than that of traditional antibody‐stained CHO cells (Figure 5C). After cells with the top 30% the fluorescence intensity was further cultured for 21 days, the mAb concentration for each subclone was measured. We have shown that both the average and the highest mAb expression level sorted by VHH‐1‐GFP is higher than that sorted by traditional antibodies (Figure 6). By monitoring expression profiles of these clones, we were able to separate and characterized clones producing high mAb levels. This result indicated that VHH‐GFP is superior for flow cytometry sorting to efficiently enrich high mAb‐expressing CHO cells compared with the traditional antibody.

In summary, recombinant anti‐Fc VHH‐GFP presents an inexpensive and liable immunoreagent for screening high mAb‐producing clones from transfected pools.

## CONFLICT OF INTEREST

The authors have declared no conflict of interest.

## Data Availability

Data openly available in a public repository that issues datasets with DOIs.
